# The Effect of Propofol plus Remifentanil for PostoperativePain and Heart Rate Management in Patients Undergoing Abdominal Hysterectomy

This article has been retracted.

**DOI:** 10.1155/2022/7646361

**Published:** 2022-07-09

**Authors:** Li Zhang, Yuping Wang, Longxin Zhang, Xiaofen Chen, Min Zhou

**Affiliations:** Department of Anesthesiology, Fujian Maternity and Child Health Hospital, Affiliated Hospital of Fujian Medical University, 18 Daoshan Road, Fuzhou 350001, Fujian, China

## Abstract

**Purpose:**

To explore the effect of propofol plus remifentanil for postoperative pain and heart rate management in patients undergoing abdominal hysterectomy.

**Methods:**

In this prospective randomized controlled study, 96 patients who underwent abdominal hysterectomy in an affiliated hospital of Fujian Medical University from April 2016 to April 2017 were recruited and randomized into the study group (*n* = 48) and control group (*n* = 48) via the random number table method. The control group received remifentanil for anesthesia, and the study group was given propofol plus remifentanil. The postoperative pain and heart rates of patients were compared between the two groups.

**Results:**

No significant difference was observed in the heart rate and adrenaline values between the two groups before anesthesia, and the study group had significantly lower adrenaline values and heart rates intraoperatively and 15 min after operation than the control group. Patients in the study group showed shorter time-lapse before independent breathing recovery, extubation, and resuscitation compared to those in the control group. The study group received less patient-controlled intravenous analgesia (PCIA) as compared to the study group within 48 h after operation. In the study group, the numeric rating scale (NRS) scores within 1 h, 2 h, 6 h, 8 h, and 12 h after operation were significantly lower than those in the control group (*P* < 0.001). Propofol plus remifentanil offer a viable alternative for postoperative pain management and stress alleviation after abdominal hysterectomy with a high safety profile. Further clinical trials are, however, required prior to clinical promotion.

## 1. Introduction

Uterine fibroid is a common female reproductive system disease, with a high prevalence in women aged 30–50 years old [1]. Abdominal hysterectomy is applicable for patients with obvious symptoms, no fertility requirements, or possible malignant changes [2]. A hysterectomy typically is performed under general anesthesia [3]. Research has indicated that postoperative stress is associated with factors such as the method of anesthesia and surgical procedures [4]. Hysterectomy requires prolonged pneumoperitoneum and Trendelenburg position, which can induce physiological changes due to increased intraabdominal pressure and consequently postoperative stress [5]. Therefore, proper anesthesia contributes to reducing postoperative pain and stress response of patients. Studies have confirmed that remifentanil is a short-acting anesthetic that takes effect after one minute of intravenous injection, lasts about 5–10 minutes, and has favorable metabolic effects [6, 7]. Remifentanil is widely used in anesthesia and is of little effect on postoperative recovery, but intraoperative dosage management is difficult [8]. Propofol is good for the induction and maintenance of general anesthesia and can balance the anesthesia dose and sedation depth, with a short half-life, rapid effect, and low toxicity [9]. However, its clinical effects are considered modest [10], and high doses of propofol can induce hypotension and momentary apnea, so remifentanil and propofol are often used in combination to enhance the effect of anesthesia [11].

Finally, 96 patients who underwent abdominal hysterectomy were recruited to evaluate the anesthetic effect of propofol plus remifentanil and its influence on postoperative pain and heart rate.

## 2. Materials and Methods

### 2.1. General Materials

In this prospective randomized controlled study, 96 patients who underwent abdominal hysterectomy in an affiliated hospital of Fujian Medical University from April 2016 to April 2017 were selected and randomized into the study group (*n* = 48) and control group (*n* = 48) via the random number table method. This study was approved by the Ethics Committee of Fujian Medical University (February 2016, 2016–02/473). All patients and their families provided written informed consent.

### 2.2. Inclusion and Exclusion Criteria

#### 2.2.1. Inclusion Criteria

Patients with surgical indications of laparoscopic total hysterectomy, with American society of anesthesiologists (ASA) [12] grades I-II; aged 18–65, and without fertility requirements were included.

#### 2.2.2. Exclusion Criteria

Patients who received the treatment in relation to analgesic in the past 14 days, with brain, heart, kidney, liver, and other organ diseases, with mental disorders such as cognitive dysfunction, and with allergies to the drugs used in this study were excluded.

### 2.3. Methods

Patients fasted for 8–12 hours before operation. After entering the operating room, patients received 10–15 ml/(kg/h) of lactated Ringer's solution (approval number: H20057482, manufacturer: Nanjing Xinfan Biotechnology Co., Ltd.) through intravenous infusion, and the dynamic electrocardiogram of the patients was closely monitored. After 2-3 minutes of oxygen inhalation, patients received 0.05–0.1 mg/kg of midazolam (approval number: H20143222, Jiangsu Jiuxu Pharmaceutical Co., Ltd) through intravenous injection, 0.08 mg/kg of vecuronium bromide (approval number: H20067266, Chengdu Tiantai Pharmaceutical Co., Ltd.), and 0.15 *μ*g·kg^−1^·min^−1^ of remifentanil (approval number: H20143314, Yichang Renfu Pharmaceutical Co., Ltd.), followed by tracheal intubation and connection to a breathing machine at 4–7 minutes after the injection. The patients then received vecuronium bromide through intravenous injection to relax muscles before operation.

The control group received remifentanil to maintain surgical anesthesia, and the study group received 4 mg–8 mg/(kg/h) of propofol and remifentanil (approval number: H20093542, Hebei Yipin Pharmaceutical Co., Ltd.) through intravenous infusion. The administration of anesthetics was discontinued at the end of the procedure. After operation, all patients received postoperative patient-controlled intravenous analgesia (PCIA) with 1 *μ*g/kg of sufentanil and 7 mg of ondansetron diluted in 100 ml of saline, with a background dose of 1.5–2 ml/kg, the self-control dose of 1 ml/time, and the lockout time of 18 min. Patients in the two groups were both treated by the same nurse and the same anesthesiologist, with the same preanesthesia, intraoperative, and postoperative treatments.

### 2.4. Evaluation Indexes

The adrenaline levels and heart rates of patients were determined in the two groups before anesthesia (D1), at 10 minutes after pneumoperitoneum establishment (D2), and at 15 minutes after operation (D3), respectively.

The time-lapse before breathing recovery, extubation, orientation recovery, resuscitation, and the frequency of PCIA within 48 hours after operation between the two groups were recorded.

The numeric rating scale (NRS) [13] was used to evaluate the physical pain of patients in the two groups at 1 h, 2 h, 6 h, 8 h, and 12 h after operation, with a full score of 10 points. The higher the score, the more severe the physical pain of patients.

Postoperative adverse reactions of patients in the two groups, including nausea, vomiting, urinary retention, and irritability, were recorded.

### 2.5. Statistical Analysis

All the data in this study were statistically analyzed and processed by the SPSS 21.0 software. The R software was adopted for sample size calculation (power = 0.8, effect size = 0.6, sig.level = 0.05); the minimum sample size was 44 cases in each group. According to the normality analysis, the continuous data in this study followed the normal distribution, so it was described in the form of mean ± standard deviation. The comparison between the groups was conducted by two independent samples *t*-test, and the comparison between multiple time points within the group was conducted by the one-way ANOVA and post hoc test. The enumeration data were described by (*n*, %) and analyzed using the *X*^2^ test. The statistically significant results were defined as *P* < 0.05.

## 3. Results

### 3.1. Clinical Data

In the control group, there were 48 patients consisting of 26 cases of primipara and 22 cases of multipara, in which there were 25 cases of uterine fibroids, 16 cases of endometriosis, 6 cases of ovarian cysts, and 1 case of other, with the average age of 52.23 ± 4.25 years and the average weight of 59.82 ± 1.43 kg. In the study group, there were 48 patients consisting of 28 cases of primipara and 20 cases of multipara, in which there were 23 cases of uterine fibroids, 19 cases of endometriosis, 4 cases of ovarian cysts, and 2 cases of others, with the average age of 52.27 ± 4.21 years and the average weight of 59.78 ± 1.41 kg. There was no significant difference in the clinical data between the two groups (*P* > 0.05).

### 3.2. Heart Rate and Adrenaline Levels at Different Times

The heart rate and adrenaline levels of patients in the two groups before anesthesia were not significantly different (*P* > 0.05), and the heart rates and adrenaline fluctuations of patients in the study group were significantly lower at D2 and D3 compared to those in the control group (*P* < 0.05), as shown in Figure 1 and Figure 2.

### 3.3. Anesthesia Resuscitation Indices

Patients in the study group showed shorter time-lapse before independent breathing recovery, extubation, and resuscitation compared to those in the control group (*P* < 0.05), as given in Table 1.

### 3.4. Frequencies of PCIA and NRS Scores

Patients in the study group had lower frequencies of PCIA as compared to the control group (*P* < 0.05). The NRS scores of patients in the study group were all significantly lower than those in the control group at 1 h, 2 h, 6 h, 8 h, and 12 h after operation (*P* < 0.05), as shown in Figure 3 and Table 2.

### 3.5. Postoperative Adverse Reactions

Patients in the study group had a significantly lower total incidence of postoperative adverse reactions compared to the control group (*P* < 0.05), as given in Table 3.

## 4. Discussion

Abdominal hysterectomy is a common surgical method for uterine fibroids [14]. Intraoperative trauma to the abdominal muscles and parietal peritoneum can cause visceral pain [15], and improper or delayed postoperative pain management may compromise postoperative recovery. Previous studies have suggested [13] that the irritability and cognitive dysfunction that patients experience after resuscitation are associated with the method and drugs used for anesthesia during surgery [16]. Appropriate stress response protects internal tissues and organs and avoids or reduces damage from various stimuli, but excessive stress response maintains tissues and organs in a state of high functioning intensity, thereby resulting in the development of many diseases [17].

In the present study, the control group received remifentanil and the study group received propofol plus remifentanil. All enrollments achieved satisfactory anesthesia effects. Remifentanil features rapid action and metabolism and good controllability. Modern pharmacological results showed that remifentanil has little effect on hemodynamics and respiratory depression in patients undergoing gynecological laparoscopic surgery with a good analgesic effect [18]. Propofol is a new, efficient, and short-acting anesthesia drug [19], conjugates with glucuronic acid and sulfate in the liver, and metabolizes rapidly into water-soluble compounds. Here, the adrenaline levels and heart rate of patients after anesthesia, at 10 minutes after pneumoperitoneum, and 15 minutes after operation were more stable compared to those in the control group. The reason may be that propofol could take effect quickly after injection, alleviate the stress response, and reduce the secretion of adrenaline and the heart rate to enhance surgical safety. Propofol protects the damaged neurons, tissues, and organs and significantly mitigates the postoperative stress response [5, 20]. The combined medication improved the safety of surgical anesthesia and reduced the occurrence of complications.

PCIA is a self-pain management method in which doctors preset the dose of analgesic drugs according to the severity of pain and the specific disease progress, and the patients were informed of the correct use of PCIA. The present study found that the frequencies of PCIA in the study group within 48 hours after operation were 7.63 ± 1.08 times, significantly lower than 16.73 ± 1.14 times in the control group. The results by Rebecca Asher et al. demonstrated that propofol plus remifentanil for total laparoscopic hysterectomy reduced the frequencies of PCIA within 2 days after operation when compared with sevoflurane (7.56 ± 0.98 vs. 16.85 ± 1.09), indicating that combined medication anesthesia is associated with favorable pain management in patients undergoing abdominal hysterectomy and accelerates the postoperative recovery. However, the following limitations still exist in this study. This study is a single-center study with a small number of patients and no blind method, which may produce bias that compromises the reliability of the research results. Future multicenter studies with a larger sample size will be carried out to provide more reliable data for clinical references.

## 5. Conclusion

Propofol plus remifentanil offer a viable alternative for postoperative pain management and stress alleviation after abdominal hysterectomy with a high safety profile. Further clinical trials are, however, required prior to clinical promotion.

## Figures and Tables

**Figure 1:** Comparison of adrenaline levels at different times. The *X*-axis represents the D1, D2, and D3, and the *Y*-axis represents the adrenaline level at different times (ng/L). ^*∗∗∗*^*P* < 0.001.

**Figure 2:** Comparison of heart rate at different times. The *X*-axis represents the times of the D1, D2, D3, and the *Y*-axis represents the heart rate at different times (beats/min). ^*∗∗∗*^*P* < 0.001.

**Figure 3:** Comparison of PICA times. The *X*-axis represents the different groups and the *Y*-axis represents the PICA times. ^*∗∗∗*^*P* < 0.001.

**Table 1:** Comparison of recovery indexes ($\bar{x}\pm s$, min).

	*n*	Breathing recovery	Orientation recovery	Extubation	Eye-opening
Study group	48	11.06 ± 1.22	17.85 ± 2.48	15.57 ± 2.14	14.24 ± 1.82
Control group	48	13.87 ± 1.36	23.01 ± 2.27	20.04 ± 2.25	16.89 ± 1.77
*t*		10.656	10.633	9.973	7.232
*P*		<0.001	<0.001	<0.001	<0.001

**Table 2:** Comparison of the frequencies of PCIA within 48 hours after operation and NRS scores at different times after operation ($\bar{x}\pm s$, scores).

Group	*n*	NRS				
		1 h	2 h	6 h	8 h	12 h
Study group	48	1.14 ± 0.09	2.05 ± 0.12	2.17 ± 0.18	1.93 ± 0.18	1.04 ± 0.06
Control group	48	2.47 ± 0.13	3.28 ± 0.09	3.38 ± 0.16	2.88 ± 0.22	2.53 ± 0.11
*t*		58.278	56.811	34.809	23.155	82.387
*P*		<0.001	<0.001	<0.001	<0.001	<0.001

**Table 3:** Comparison of postoperative adverse reactions (*n* (%)).

Group	*n*	Vomiting	Urinary retention	Irritability	Nausea	Total incidence
Study group	48	1 (2.08%)	0 (0.00%)	2 (4.17%)	1 (2.08%)	8.33% (4/48)
Control group	48	2 (4.17%)	2 (4.17%)	4 (8.33%)	4 (8.33%)	25.00% (12/48)
*χ* ^2^						4.800
*P*						0.028

## Data Availability

No data were used to support this study.
